# Legal Early Warning of Public Crisis in Network Public Opinion Events Based on Emotional Tendency

**DOI:** 10.1155/2022/6367295

**Published:** 2022-08-23

**Authors:** Zhijuan Ni

**Affiliations:** School of Political Science and Law, Weifang University, Weifang, Shandong 261061, China

## Abstract

At present, China is in the period of social transformation, and social contradictions are gradually prominent. The research on NPO (network public opinion) emergency warning methods is gradually increasing. Some existing laws and regulations are abstracted and principled in content, lacking specific implementation rules and corresponding supporting measures, especially the legal rules of emergency administrative procedures. Therefore, the legal early warning model of NPO public crisis is based on emotional dimension content, NPO emotional characteristics, emotional dimension elements, and machine learning classification algorithm to construct text ET (emotional tendencies) classifier, which can be used to make ET judgment on text data. The results show that after PSO (particle swarm optimization) algorithm optimization, the precision, recall rate, and micro-average are significantly improved, and the precision is increased by nearly 14% and 80%. The conclusion shows that using PSO optimization parameters improves the classification effect of the classifier, and a better NPO crisis early warning model can be obtained.

## 1. Introduction

With the rapid popularization of the Internet, big data information is sprouting, and various NPOs (network public opinions), including Weibo, have gradually become the comprehensive carriers of many netizens' thoughts, opinions, and emotions. Internet public opinion often contains the personal emotions of the sender of public opinion, which will affect the public opinions of other netizens. If these emotions are not paid attention to and guided in time, they will lead to unexpected events and bring negative impacts to the society. The public crisis of NPO event is the most direct threat in the field of urban public security, which will often enlarge the scope and harm the degree of the crisis due to its expansion effect and chain effect [1]. The pre-control function of public crisis is to make a corresponding diagnosis after monitoring, identification, and evaluation, to determine whether to take corresponding pre-control countermeasures and how to take corresponding countermeasures. The prior information corresponding to a planning countermeasure system can establish early prevention and control.

When there is an emergency, the news media are rushing to follow up and report, and the public is informed of the situation through a variety of channels. This is then followed by comments, which can be for or against, emotional or rational, enthusiastic and positive, or irrelevant, like mushrooms after rain. Wang et al. proposed a crawler method that divided web pages into topic blocks and was based on topic-related concepts. The results in practice demonstrate that this approach works well for gathering data on public opinion [2]. According to the majority of two-character Chinese words, Sokhey et al. proposed the two-character hash system to significantly increase word segmentation speed [3]. This was done while maintaining the space complexity of the traditional word segmentation algorithm dictionary. A new dictionary structure with a three-level index has been proposed by Zhang et al., which shortens the time it takes to match words in the segmentation text with words in the dictionary. This structure expands the hierarchy based on the secondary index and further improves the positioning efficiency of words in the dictionary. Using a semi-supervised learning approach and a mixed statistical model of topic tendentiousness, Scott-Weaver calculated the article's overall ET (emotional tendentiousness) [4]. By examining unfavourable words, adverbs, context, and other relevant elements, Ekengren and Oscarsson created an emotional dictionary that they then used as a benchmark to assess ET [5]. The government can only know the public opinion quickly, respond quickly and appropriately to the situation, and maintain social stability by quickly obtaining these public opinion data from the Internet.

NPO refers to the interwoven sum of various attitudes, feelings, and opinions expressed and communicated by people through the Internet [6]. The Internet provides a virtual environment, and the randomness and permeability of information release make nonprofit organizations prone to complex situations where rational and irrational elements are intertwined. At present, the difficulties in the investigation of nonprofit organizations are mainly concentrated in two aspects. How to establish a perfect judgment mechanism is the research of forecasting methodology. Public legal early warning of crisis is the only way for China to develop public crisis management at the international level. It can show the government's emergency crisis management ability and enhance the government's credibility; provide a richer and more accurate theoretical and methodological basis for NPO classification monitoring and crisis early warning; and lay a theoretical foundation for the further development of related research, which has certain reference value.

### 1.1. The Main Innovation Lies in the following Aspects

1. In this study, NPO information emotional dimension is placed in the space system for the first time, and its internal comprehensive action mechanism is comprehensively considered. A series of new concepts is defined in the professional research field, and NPO information emotional dimension space theory is put forward and enriched.
2. The key of public opinion analysis lies in judging the ET nature of public opinion data and correctly distinguishing positive public opinion from negative public opinion. In this article, the vector space model is used to represent the text, and the feature extraction technology is combined with the TF-IDF algorithm to adjust the emotional weight and give words emotional features.

### 1.2. Content Structure of the Article

The rest of the article is organized as follows: Section 2 introduces the associated legal early warning technologies of public crisis in network public opinion events.  Section 3 outlines the specific procedures and application of this study. The superiority and viability of this research model are confirmed in Section 4. The full text is summarized in Section 5.

## 2. Related Works

### 2.1. NPO Research

NPO is the extension of public opinion in cyberspace, and it is the sum of all kinds of feelings, wishes, attitudes, and opinions held on various public issues that are concerned or closely related to their interests in a specific historical stage and social space. In short, we can think that public opinion refers to the expression and collection of people's social ideas, while NPO is the expression of online public opinion, which is composed of netizens, social public affairs, and netizens' will.

Turner found that the leader of online public opinion is usually a person with great influence in the society, and his opinions usually spread in the network at a very fast speed and have great influence [7]. Gearhart et al. thought NPO is a special expression of social public opinion on the Internet, and it is the opinions of people on specific social issues with their own inclination and influence [8]. Eveland et al. thought that there is collective psychology in the process of NPO spreading, which makes the opinions of individual netizens be influenced and converge [9]. Mjrg pointed out that in order to effectively control NPO, we must improve the Internet management rules, make the network information transparent, strengthen the government's guiding role in public opinion, and improve people's quality [10].

Vreese used Markov chain to analyze and estimate the heat trend of NPO, and the core is to divide the state space and construct the state transition matrix [11]. Ning et al. analyzed and predicted the long-term development trend of new events according to the model of the class to which the new events belong [12]. Its disadvantage is that the prediction performance depends entirely on the results of hierarchical clustering, and the objectivity and comprehensiveness of the clustered corpus will affect the clustering effect, thus affecting the prediction accuracy. Wang et al. have shown through research that personal opinions and their roles in the public opinion environment are the major causes of public opinion, while group emotions are the important decisive factors in the change of public opinion [13]. Liu et al. thought that they can quickly process a large amount of NPO information, observe the development trend of public opinion according to the method of rough classification and transcendence, and put forward corresponding strategies to keep a stable information environment running steadily [14].

### 2.2. ET Research Status

The research direction of ET analysis is a hot spot in the field of text mining. There are many knowledge and technical points involved. From the perspective of teleology, text ET analysis technology requires computers to recognize human ET descriptions. At a deeper level, computers are required to understand human ET. The ultimate goal of ET research is to make computers understand the ET of others and computers like people.

Weibo is used as the corpus, but the difference is that Wang first constructed an emotional dictionary for Chinese Weibo and used emotional words as text features. After the corresponding text preprocessing, Wang calculated the weighted values of all emotional words in Weibo, thus obtaining ET [15]. After collecting the corpus, Coa et al. first extracted the subjective text by spectrum technology, removing the objective text that had no influence on text classification and then classified the text by the method of combining active learning with ensemble learning [16]. Mittelstaedt et al. first proposed a spam comment detection method based on clustering for effective filtering of spam comments and then proposed a new text feature representation method, namely feature selection based on nonnegative matrix decomposition. Finally, several feature selection methods were compared with the existing classifier, and the experiment proved that this method has higher accuracy [17].

ET analysis of words is the premise and foundation of text ET analysis. Yuan finds out subjective sentences by using the similarity calculation method and multiple NB (naive Bayes) classifier [18]. Wu et al. used the times of words appearing in the article as weights and used NB, maximum entropy, and SVM (support vector machine) to judge whether a comment was positive or negative [19]. A text classification model based on SVM is implemented, and a new algorithm is proposed. Compared with other algorithms used before, the accuracy of this algorithm is slightly reduced, but it improves the efficiency to a great extent, and it has great application significance for text classification in reality.

## 3. Methodology

### 3.1. Emotional Dimension Analysis of NPO Information

The complexity and correlation between the data are high, and NPO has a lot of data. How emotional information is organized and evaluated in NPO will greatly affect how well the emotional semantics of public opinion are recognized and comprehended. Information about public opinion is not subject to ET analysis in semantic analysis technology. Many unique pieces of information about the public's opinion, whether favourable or unfavourable, are determined by the speed and complexity of information changes in the big data environment. Subversive emotional changes will occur as a result of the unanticipated stimulation of a particular public opinion environment, which is crucial public opinion data. The evolution of forwarding and commenting is inextricably linked to emotional concern and preference in the process of moving from recessive public opinion to dominant public opinion. This is especially true in the social network of recessive public opinion.

The widely employed techniques for text trend analysis can be broadly categorized into two groups: classification algorithms based on emotion word matching tables and classification algorithms based on machine learning. This article proposes a machine learning classification algorithm based on emotion weight adjustment, performs ET analysis on the text data, and attempts to improve the accuracy and the most persuasive text direction judgment through a thorough analysis of the aforementioned two methods, combining the benefits and drawbacks of the two methods. Text trend analysis based on a machine learning classification algorithm generally includes six steps: selecting training sample data, building a text representation model, extracting text features, training classification model, and selecting an appropriate classification model for ET classification and trend analysis, as shown in Figure 1.

The text representation model, for example, transforms unstructured text data into structured data that computers can comprehend and learn; not every word or character is examined for features. The ranking models should be compared in accordance with the machine learning ranking algorithm evaluation indices, the benefits and drawbacks of each ranking algorithm should be made clear, and the ranking models that are unsuitable for the practical application of public opinion analysis should be disregarded. High-level emotion, intermediate emotion, low-level emotion, and irrelevant emotion are the four categories used in this model to categorize the emotional level of NPO information. There are various stages of development and layer jumps. Extroverted emotions can result from advanced emotions, such as expressing intense care and concern for the opinions of the public that are for the better, expressing a strong sense of duty for the opinions of the public that are for the worse, and producing moderately strong or excessively aggressive emotional reactions.

The weight of words in a vector is no longer a simple word frequency, but the word frequency multiplied by the inverse of the text frequency, that is TF-IDF (term frequency-inverse document frequency). The weight formula of the TF-IDF algorithm is:

(1) $$\begin{array}{c} \omega_{ij}=TF_{ij}\times IDF_{i}=\frac{n_{ij}}{\sum_{k}n_{kj}}\times \;\log\left(\frac{N}{DF_{i}}\right). \end{array}$$

Space is composed of different dimensions, dimension lines form different shapes, and the part inside dimension lines is space. NPO information emotion has the psychological three-dimensional structure of the essential development of public opinion information movement, which is used to represent the generation and interaction of public psychology, emotion, and consciousness of public opinion participants. Any element of information is centered on subspace. Although there are differences between points, these differences are constantly balanced, which is the essential feature of NPO information emotional dimension space. Here, the data opinion points are expressed as follows:

(2) $$\begin{array}{c} P=\left(r,\theta ,\varphi \right)\left[\phi \right], \end{array}$$

where *r* is the distance from the information emotion element *P* to the origin of the coordinate system, and its measured value is a nonnegative real number, and *θ* ∈ [0, *π*], *φ* ∈ [0,2*π*] and *ϕ* are edge coordinate values.

NB classifier has been used for machine learning problems such as classification for a long time. The ratio of joint probability and conditional occurrence probability is obtained by the product of inverse conditional probability and inverse conditional occurrence probability. The formula is as follows:

(3) $$\begin{array}{c} P\left(A|B\right)=\frac{P\left(B|A\right)*P\left(A\right)}{P\left(B\right)}, \end{array}$$

where *P*(*X*) refers to the probability corresponding to the event *X*. For a test document to be classified, after it is represented as a vector space model, based on the assumption of independence between words, the posterior probability of the vector under each category is calculated, and the category corresponding to the highest probability event is selected as the classification result.

Obviously, the construction of the classification model is the most important link in text classification, and the quality of the classifier will directly affect the classification effect. Among all machine learning methods, Gaussian process is a relatively mature classification and regression prediction algorithm.

Gaussian process is completely determined by the mean function and covariance function. As long as the mean function *m*(*x*) and covariance function *K*(*x*, *x*′) are determined, this Gaussian process will be determined. The function is expressed as:

(4) $$\begin{array}{c} f\left(x\right)∼gp\left(m\left(x\right),K\left(x,x^{\prime }\right)\right). \end{array}$$

The hyperparameters of traditional Gaussian processes are determined by conjugate gradient method, which is obtained by maximizing the log-likelihood function of training samples. Because the conjugate gradient method has some disadvantages, such as the number of iterations is difficult to determine, the dependence on the initial value is strong, and the local minimum value is easy to drop, etc., this article uses PSO (particle swarm optimization) algorithm to improve the Gaussian process. In order to improve the convergence speed and solution quality of the basic PSO algorithm, the inertia-weighted PSO algorithm, that is the improved speed updating formula, is used, as shown in the following expression:

(5) $$\begin{array}{c} v_{id}=w\cdot v_{id}+c_{1}\cdot \text{rand}\left(\right)\cdot \left(P_{id}-x_{id}\right)+c_{2}\cdot \text{rand}\left(\right)\cdot \left(P_{gd}-x_{id}\right), \end{array}$$

where *c*_1_, *c*_2_ are positive acceleration coefficients, *c*_1_ expresses the dependence of particles on their own memory, *c*_2_ determines the influence of other particles in the particle group on themselves, and rand() is a random number with a uniform distribution between 0 and 1, which is used to simulate slight fluctuations in group behavior in nature, *P*_*id*_ is the *d*-dimensional component of individual extremum, and *P*_*gd*_ is the *d*-dimensional component of global extremum.

This information sharing mechanism is more conducive to the rapid convergence of the algorithm. Therefore, the PSO algorithm is used to automatically search the optimal hyperparameter of the Gaussian process in the sample training process, and a Gaussian process algorithm based on PSO is formed.

### 3.2. Realization of Legal Early Warning of NPO Event Public Crisis

At the moment, China's one-stop legal standards for public crisis management are primarily focused on accident- and disaster-type public crises, with little involvement in other areas. For instance, the laws governing national security crisis management, such as the National Defense Mobilization Law and the Terrorism Crisis Management Law, are deficient. From a practical standpoint, it is necessary to further enhance the fundamental social conditions, such as public awareness, recognition, adaptability, degree of cooperation, and social psychological conditions, of the legal framework for public crisis management. The highest administrative organ of the state has the authority to authorize and delegate the exercise of the law. Implementing the rule of law reservation can essentially ensure the supreme legislative authority's unrestricted decision-making authority over important matters of national concern as well as the legitimate protection of citizens' rights.

The public can comment on emergencies as a concentrated expression of social problems and contradictions through the network platform, and different users can discuss with one another. Emergencies and NPO are closely related through frequent information exchange. New social problems and emergencies, possibly even serial emergencies, will emerge concurrently with the NPO's ongoing spread, making it more challenging for the government to address them. Because of these characteristics of emergencies, NPO emergency warning is more important and difficult [7]. For public interest emergencies, there may be tens of thousands of comments on the Internet, and it is impossible to collect all comments. According to the timing of netizens' comments and the randomness of their content, the number of samples to collect comments after the event can be determined according to the influence of the event and the attention of the network [9]. One person's ET can greatly affect another person's ET. After an emergency of public concern, personal online comments will have different degrees of influence on the emotions of netizens who are concerned about the incident, and then the affected netizens will make the same or similar comments, thus affecting more people.

In my opinion, we should establish public crisis early warning laws and regulations for nonprofit organizations based on foreign experience, perfect the current laws and regulations, and then incorporate them into the public crisis management of all different types of nonprofit organizations. The government must harmonize policies and systems in order to provide early warning of crises. Power and responsibility, a clearer understanding of the precise duties of pertinent departments and organizations, improved information sharing for early warnings, and realization of public crisis early warnings for nonprofit organization events are all required by law. Therefore, efforts should be made to improve internal robustness, on the one hand, and reduce the arrival rate of external police sources when an incident occurs during the public crisis management process of nonprofit organizations on the other hand. Based on this, Figure 2 illustrates how an early warning model of NPO public crisis events was built in a law.

The government and social management departments should set up pertinent databases and early warning and evaluation mechanisms to analyze and monitor the number and rank of police sources when there are enough police sources in the system and the NPO incident turns into a public crisis. To ensure the accuracy of the evaluation, the early warning evaluation mechanism should be improved; a data analysis mechanism should be set up; evaluation procedures and guidelines should be created; and early warning personnel should be directed in filtering, organizing, and processing the original data. The establishment of an emergency command center, whose main duty is to coordinate the work of relevant departments, logically dispatch emergency resources, and make some crucial decisions, is one of the solutions put forth for specific problems at the business level in conjunction with the emergency plan.

The basis of ET value calculation is an emotional dictionary, and representative *k* pairs of reference words are selected, and each pair of reference words includes a commendatory word and a derogatory word. *p* denotes a commendatory reference word, *q* denotes a derogatory reference word, and the formula for calculating the vocabulary ET value of Orient(*w*) is as follows:

(6) $$\begin{array}{c} \text{Orient}\left(w\right)=\sum_{i=1}^{k}\text{Sim}\left(p_{i},w\right)-\sum_{j=1}^{k}\text{Sim}\left(q_{i},w\right). \end{array}$$

The value of Orient(*w*) represents that degree of praise and criticism of the word *w*, and Sim(*q*_*i*_, *w*) represents the semantic similarity between the word *w* and the reference word.

Considering the influence of short text and long text on the absolute weight of word frequency, the absolute weight of word frequency can be normalized by the length of text, that is the normalized weight of word frequency. Therefore, this article adopts the TF-IDF weighting method, which not only considers the local word frequency of feature words, but also considers the word frequency in the global text. In this work, the formula is improved, and the factor of ET value of emotional words is added. The improved weight calculation formula is as follows:

(7) $$\begin{array}{c} W_{ik\left(\text{new}\right)}=VET_{\text{new}}\left(t_{k}\right)\cdot \frac{tf_{ik}\cdot \;\log\left(N/n_{k}+0.01\right)}{\sqrt{\sum_{i=1}^{n}{\left(tf_{ik}\right)}^{2}\cdot \;\log^{2}\left(N/n_{k}+0.01\right)}}, \end{array}$$

where *f*_*ik*_ represents the frequency of feature *t*_*k*_ appearing in document *d*_*i*_, *N* represents the total number of documents in the training set, and *n*_*k*_ indicates the number of documents with feature *t*_*k*_. *VET*_new_(*t*_*k*_) is the vocabulary ET value.

At the same time, the risk function is added to the SVM public opinion emotion classification algorithm combined with regression prediction, as shown in the following formula.

(8) $$\begin{array}{c} R_{\text{reg}}=\frac{1}{2}{\left\|w\right\|}^{2}+C*R_{\text{emp}}^{\varepsilon }\left[f\right], \end{array}$$

where ‖*w*‖^2^ refers to a descriptive function about public opinion emotion classification, *C* is a constant, and *f*() refers to the model complexity of public opinion emotion classification algorithm. The insensitive loss function *ε* is introduced to improve the function. After improvement, the function is expressed as follows:

(9) $$\begin{array}{c} {\left|y-f\left(x\right)\right|}_{\varepsilon }=\left\{\begin{array}{cc} 0, & \left|y-f\left(x\right)\right|\leq \varepsilon ,\\ \left|y-f\left(x\right)\right|-\varepsilon , & \text{other}. \end{array}\right. \end{array}$$

The whole process of NPO's emergence, formation, and development is based on the network, and the information involved is scattered and embedded in massive data, including new online media such as news websites and online communities, which contain a large amount of potential information related to the subject. It is necessary to construct the measurement pattern set and attribute set, determine each threat target as an alternative pattern, and then combine multiple threat targets into a decision pattern set [8]. Then it is necessary to establish a decision matrix and a target threat estimation model. Finally, the degree of target threat is classified by approaching the ideal classification method of each scheme. The whole public opinion crisis prediction and early warning system are mainly divided into three modules as shown in Figure 3.

Pre-control and crisis management, according to the prediction and early warning model results of Module 2 and Module 3, can put forward corresponding solutions and suggestions. The knowledge base of this module consists of case base and solution set. If feasible, it can directly solve the crisis and input the corresponding solutions into the knowledge base. Otherwise, a new solution is deduced by reasoning technology and knowledge is inputted.

## 4. Experiment and Results

In case of emergency, the actions of relevant departments are correct. After the incident, the relevant departments announced that they would take it seriously according to law, which played a role in stabilizing netizens' emotions to a certain extent. First, feedback from netizens should be collected and then where the netizens are concentrated should be analyzed. Second, the warning level should be determined. Finally, according to the analysis results, specific guidance from ET should be taken. The number of samples collected this time is 20 related Weibo, and each Weibo has 40 comments. The results are shown in Figure 4.

We should adopt the yellow warning level 2 because 36.4% of the public are of the opinion that social harmony is not important. Considering the analysis above, the following actions are possible: the matter will be handled in accordance with the law. It demonstrates that the staff is also average citizens and that their conduct does not speak for the organization or the government and cannot serve as a representative of either. Legal action is taken against anyone who knowingly encourages netizens to despise wealth and defame the government. From the test corpus, we must extract as many words that express emotion as we can and determine their polarity. Note that when degree or negative adverbs are used to modify words with strong emotional connotations, the original emotional polarity and intensity are altered. The combination and output of modifiers and emotive words is therefore required.  Figure 5 depicts the trend of improving evaluation times and increasing emotional word recognition accuracy.

We can see that whether it is the ET word judgment model based on NB classification or the ET word judgment model in this article, the accuracy of its recognition and judgment gradually decreases with the increase of evaluation times, but the latter decreases with the increase of evaluation times, and the speed is much slower, which indicates that the method adopted in this work has certain stability. The comparative experimental data of this text sentiment classification model and SVM text sentiment classification model are shown in Table 1.

In this article, the model text ET discrimination accuracy is about 86%, the recall rate is about 82%, and the F value is about 79%. Compared with the text ET parsing model of SVM, it is obviously improved. Especially the text sentiment classification model is superior to the low value of the traditional text ET analysis model in terms of retrieval rate, which is close to the accuracy value. It holds that the emotional words or phrases in the text are independent of each other, but just as the emotional computing model of the text based on polarity accumulation says, the ET of the text must also reflect the emotional evolution process of the author.

A classifier is built and trained according to the process of building a classifier above. After the training, each part of the test corpus is tested separately, and all the above processes are tested in MATLAB. After the experiment, precision, recall rate, and micro-average are calculated according to the experimental results, which are shown in Figure 6.

As can be seen from the above pictures, the precision, recall, and micro-average of the Gaussian process are obviously improved after being optimized by the PSO algorithm (there are very few low phenomena), among which the accuracy is improved by nearly 14% and nearly 80%. It shows that parameter optimization with PSO plays an important role in improving the classification effect of the classifier. ET research can be divided into different levels according to different tasks. In previous studies, the most widely used strategy is to use manually compiled dictionaries for identification. Obviously, in the network environment, a large number of new words are derived, and some old words are discarded, which cannot be solved by a dictionary. This document also verifies the effect of the final result. The standard answers in the evaluation corpus were used as the scoring basis. Finally, the final evaluation results are compared (Table 2).

It can be seen that the strategies put forward in this work are close to the best results among all participating teams. The strategy proposed in this article is based on a semi-supervised statistical machine learning method. Except for simple Chinese semantic units and simple thesaurus, it is not easy to achieve such a result without the application of a large-scale prior corpus, and the whole research work has certain practical application value. The division of NPO information emotional dimension subspace can be determined by membership frequency, and the data distribution and spatial characteristics of each subspace of NPO information emotional dimension are further analyzed. The spatial domain of NPO information emotional dimension is clustered, each cluster is represented by the set A1, A2, A3, and A4 of each subspace, and the membership frequency/number of experiments is the membership frequency of each cluster (Figure 7).

It can be seen that the subspace of the instinctive layer is nondirectional emotional information, which has strong implicit features, and the emotional arousal dimension is activated or close to zero. Because of its strong judgment, the information coverage will be relatively wide. In the gathering areas with high concentration, the early warning degree of public opinion crisis in this area is high, and the information and emotional items with high concentration rate also have certain characteristics of spatial aggregation and contact with the public. Session subspace belongs to the emotional space segment with the separation of internal and external concepts, and its membership frequency is low. Reflective subspace belongs to the advanced emotional category of social level, and its extroversion is more obvious, and its subordinate frequency of emotional data is the most concentrated.

Figure 8 is a schematic diagram of the prediction result obtained by using the improved neural network model to predict the number of network responses. The experimental results show that the neural network model has superior performance in predicting NPO development trend. ET analysis model combined with expression attention mechanism and nonemphasis expression attention mechanism improves the accuracy of sentiment analysis of public opinion texts by 4.01%, which shows that the relationship between expressions and texts is in the emotional polarity of comment texts.

Public crisis early warning is not just a mechanism; it is also deeply ingrained in people's social consciousnesses and cultural norms. They should attack as the appropriate personnel involved in public crisis early warning, so that they can carry out their duties more effectively. Early crisis detection affects social harmony, stability, and the safety of people and their property. We must promptly evaluate training in order to be serious and ensure its effectiveness and quality. In terms of training content, it is essential to switch from conventional book training to actual combat training with strong practical ability as the main training, consistently conduct actual combat simulation and case analysis, accumulate early warning experience, and inspire the team.

## 5. Conclusions

Unexpected events frequently become the center of attention and start a chain reaction of related events. The development of a public crisis management system's legal early warning system is the first line of defense and a representation of the stability of a civil society. By contrasting the ET classification judgment effects of various emotional word weight calculation methods and machine learning classification algorithms, this article, which is based on the theory of the emotional dimension, proposes a classification algorithm based on emotional word weight. It also identifies the crucial NPO change turning point and focuses on analyzing the negative direction and the causal relationship of public opinion formation in each stage. The trend of NPO information emotion is predicted based on the coordinates and separations of the information emotion elements in the NPO information emotion space, which serves as a useful guide for accurately locating NPO. The outcomes of the experiment demonstrate that neural networks are more practical and efficient in providing a legal early warning of NPO public crisis.

## Figures and Tables

**Figure 1:** Flow chart of text tendentiousness analysis.

**Figure 2:** Legal early warning model of NPO event public crisis.

**Figure 3:** NPO prediction and early warning system architecture.

**Figure 4:** Public opinion data collection and statistics.

**Figure 5:** Trend of the accuracy of emotional polarity discrimination.

**Figure 6:** Comparison of evaluation indexes of each part of the optimized training corpus.

**Figure 7:** Membership frequency value of NPO information emotional dimension subspace.

**Figure 8:** Predicted values and errors obtained by the model.

**Table 1:** Comparative experimental data of text sentiment classification model.

Model	Object	Accuracy (%)	Recall (%)	F value (%)
Model of this article	Emotional words	0.863	0.824	0.796
	Words + emotional phrases	0.842	0.816	0.791

SVM	Emotional words	0.801	0.799	0.768
	Words + emotional phrases	0.812	0.781	0.753

**Table 2:** Phrase extraction result.

Result sequence	Macro-average			Micro-average		
	Accuracy (%)	Recall (%)	F value (%)	Accuracy (%)	Recall (%)	F value (%)
IG	8.124	7.769	7.968	10.014	7.966	9.068
Average	5.536	5.063	4.665	7.638	6.325	6.201
Best	8.146	10.012	8.714	11.741	10.217	10.251

## Data Availability

The data that are used to support the findings of this study are available from the author upon request.
